# Exponential Time Differencing Method for Studying Prey-Predator Dynamic during Mating Period

**DOI:** 10.1155/2021/2819145

**Published:** 2021-09-21

**Authors:** Noufe H. Aljahdaly, H. A. Ashi

**Affiliations:** ^1^Department of Mathematics, Faculty of Sciences and Arts-Rabigh Campus, King Abdulaziz University, Jeddah, Saudi Arabia; ^2^Department of Mathematics, Faculty of Science, King Abdulaziz University, Jeddah 21589, Saudi Arabia

## Abstract

This paper addresses a first numerical simulation to the nonlinear dynamic system of equations that describes the prey-predator model at the predator mating period. Some male species accompany the females during the mating period. In this case, both male and female feed on the same prey. The presented work shows the numerical solution for this specific case of the prey-predator mathematical model via an exponential time differencing method. In addition, the paper provides the biological implication of the solution.

## 1. Introduction

Many applications and phenomena in physics, biology, the medical field, and other fields can be described as a mathematical model in order to understand or predict the dynamic of these phenomena or applications [1–3]. The prey-predator model is a famous biomathematical model that has been investigated widely to study the dynamic of the ecology system and an intersection between prey and predator [4]. The Lotka-Volterra model is known as the predator-prey model for the study population process [5–7]. The model has been studied when considering the influence of diseases [8], prey refuge [9], food chain [10], or competitive populations [11]. The model also was developed to study the intersection between two different populations of predators and one prey [12, 13]. Recently, the model was modified to study the intersection between two predators from the same species (female and male) and one prey. In some species, the male stays with the female all the time, and they feed together at the mating period. This model is given as follows [14]:

(1) $$\begin{array}{c} u_{t}=a_{1}u-a_{2}u^{2}-a_{3}uv-a_{4}uv^{2},\\ v_{t}=D_{2}\left(\Delta v\right)+a_{3}uv-a_{5}v-a_{6}v^{2}+a_{4}uv^{2}, \end{array}$$

where *u* and *v* are the total numbers of prey and predator, respectively. *a*_1_ is the prey's growth rate. *a*_2_, *a*_3_, and *a*_4_ are the prey's decay rate due to competition on food supply between the male and the female, between one predator and one prey, and between two predators and one prey, respectively. *a*_5_ is the mortality rate for the predator. *a*_6_ is the decay rate of the predator due to competition on the food supply between the male and the female. *D*_2_ is the predator's diffusion term. In Reference [14], the system (1) was rescaled and became a dimensionless nonlinear system as follows:

(2) $$\begin{array}{c} U_{t}=U-U^{2}-UV-UV^{2},\\ V_{t}=V_{XX}-k_{2}k_{1}V-k_{1}V^{2}+k_{1}VU+k_{1}UV^{2}, \end{array}$$

where $k_{1}=\sqrt{a_{4}a_{1}}/a_{2}=a_{3}/a_{2}$ and *k*_2_ = *a*_5_/(*a*_1_*k*_1_).

The mathematicians put forth more effort in the computational field to improve different techniques to be able to find the consistent solutions for realistic applications, for example, the geometric-qualitative method, semiapproximate method, qualitative method, numerical method, and analytical method. Analytical methods generate different solutions based on many factors such as used ansatz. There are many methods to obtain the analytical solutions such as the (*G*′/*G*^2^)-expansion approach [15] and the direct algebraic method [16–19]. They are able to obtain the solutions without an initial condition. Each method can introduce new solutions to the system. The solutions of system (2) were found by two analytical methods, the (*G*′/*G*^2^)-expansion approach and the direct algebraic method [15]. Since the analytical methods give different solutions, it is difficult to determine which solution predicts the applications. On the other hand, the numerical method for the initial value problem is the method that finds the approximate solution and converges to only one solution based on the initial condition that is obtained from the application, for example, the finite difference method [20–22], Adomian decomposition method (ADM) [23], Laplacian Adomian decomposition method (LADM), multistage differential transform method [24, 25], and exponential time differencing method [26]. The numerical solution for system (2) will be introduced in this paper via the exponential time differencing method since the method is fourth-order accurate and is not local convergent comparing to ADM or LADM. The results either determine which analytical solution that predicts the problem or find a new solution.

The paper is organized as follows: the next section presents the numerical results and the scheme of the used method, the third section discusses the numerical solution from the biological perspective, the fourth section is a comparison with the previous studies for the aforementioned model, and the last section is the summary of our analysis and results.

## 2. Numerical Simulation

In this section, we give the approximate numerical solution of system (2). First, the system is discretized in space utilizing the Fourier spectral method. Hence, we obtain the following system of ordinary differential equations (ODEs) that depends only on time:

(3a) $$\begin{array}{c} \frac{d{\hat{u}}_{k}\left(t\right)}{dt}={\hat{u}}_{k}\left(t\right)+{\hat{F}}_{k}\left({\hat{u}}_{k}\left(t\right),{\hat{v}}_{k}\left(t\right),t\right), \end{array}$$

(3b) $$\begin{array}{c} \frac{d{\hat{v}}_{k}\left(t\right)}{dt}=c{\hat{v}}_{k}\left(t\right)+{\hat{G}}_{k}\left({\hat{u}}_{k}\left(t\right),{\hat{v}}_{k}\left(t\right),t\right), \end{array}$$

where the parameter *c* = *k*^2^ − *k*_2_*k*_1_ is associated to the linear part, *k* represents the wave numbers, both terms

(4) $$\begin{array}{c} {\hat{F}}_{k}\left({\hat{u}}_{k}\left(t\right),{\hat{v}}_{k}\left(t\right),\left.t\right)\right)=fft\left(-U^{2}\left(t\right)-U\left(t\right)V\left(t\right)-U\left(t\right)V^{2}\left(t\right)\right),\\ {\hat{G}}_{k}\left({\hat{u}}_{k}\left(t\right),{\hat{v}}_{k}\left(t\right),\left.t\right)\right)=k_{1}fft\left(-V^{2}\left(t\right)+U\left(t\right)V\left(t\right)+U\left(t\right)V^{2}\left(t\right)\right), \end{array}$$

represent the nonlinear forcing term, and fft is the MATLAB command that represents the fast Fourier transform (FFT).

Second, we integrate the obtained uncoupled system of ODEs (3) in time with the aid of the fourth-order exponential time differencing method ETD4RK [27–29]. Applying the ETD4RK method to (3b) takes the formula

(5) $$\begin{array}{c} a_{k,n}={\hat{v}}_{k,n}e^{c\Delta t/2}+\left(e^{c\Delta t/2}-1\right)\frac{{\hat{G}}_{k,n}}{c}, \end{array}$$

(6) $$\begin{array}{c} {\hat{v}}_{k,n+1}={\hat{v}}_{k,n}e^{c\Delta t}+\left(\left(c^{2}\Delta t^{2}-3c\Delta t+4\right)e^{c\Delta t}-c\Delta t-4\right){\hat{G}}_{k,n}+2\left(\left(c\Delta t-2\right)e^{c\Delta t}+c\Delta t+2\right)\left(\hat{G}\left(a_{k,n},t_{n}+\frac{\Delta t}{2}\right)+\hat{G}\left(b_{k,n},t_{n}+\frac{\Delta t}{2}\right)\right)+\frac{\left(\left(-c\Delta t+4\right)e^{c\Delta t}-c^{2}\Delta t^{2}-3c\Delta t-4\right)\hat{G}\left(C_{k,n},t_{n}+\Delta t\right)}{c^{3}\Delta t^{2}}, \end{array}$$

where Δ*t* represents the time step (a similar formula is obtained when applying the ETD4RK method to (3a) with *c* = 1).

The time integration starts with initial conditions (taken from [30]) given by

(7) $$\begin{array}{c} {\hat{u}}_{0}=\frac{6}{35}-2\times 10^{-7}\left(x-225\right)\left(x-675\right),\\ {\hat{v}}_{0}=\frac{116}{245}-3\times 10^{-5}\left(x-450\right)+180\times 10^{-4}. \end{array}$$

The results of our experiment are shown in figures.

The solution is stable at $0\leq k_{2}\leq \left(1+\sqrt{5}\right)/2$ based on the stability analysis in Reference [14]. A numerical solution is produced in Figure 1 for different value of *k*_2_. We realized that solutions are changed with *k*_2_. When *k*_2_ = 1.5, *U* increases while *V* decreases until they reach the steady state. For *k*_2_ = 0.1, the solution is periodic. The parameter $k_{2}=\left(a_{2}a_{5}\right)/\left(a_{1}\sqrt{a_{4}a_{1}}\right)=\left(a_{5}a_{2}\right)/\left(a_{1}a_{3}\right)$ has direct relation with *a*_5_ and *a*_2_ and negative relation with *a*_1_, *a*_3_, and *a*_4_.

## 3. Biological Relevance of the Solution

A new term in the studied model is *a*_4_*v*^2^*u*. Thus, the numerical solution is used to study the effect of this term on a traditional prey-predator model. The solution of the traditional model is an undamped oscillation, and Lotka explained this behavior because of the law of mass action [5], while the presented model (2) has an oscillation solution with small *k*_2_ at a bounded space and the solution converges to the steady state out of this space, because *a*_4_*v*^2^*u* is related to the interaction between prey and two predators at the mating period which disappears after this period and also happens in a specific location where the predators give birth.

The large rate of *a*_4_ indicates that the predators feed on a large amount of prey in this period, which lead to a large size of the predator population than the prey population. This is not an optimal dynamic of population to live normally (see Figure 2 when *a*_4_ = 10). Therefore, the predator population will decrease because of absence of a food source, while the prey population will grow again. The new term *a*_4_*v*^2^*u* has more effect than *a*_3_*uv* to decay the prey population as we see by comparing Figures 3 and 2.

## 4. Connection with the Previous Studies

The analytical solutions of Equations (2) was found by Aljahdaly and Alqudah [31] using (*G*′/*G*) and the generalized auxiliary equation [15]. The solutions are *U*(*x*, *t*) and *V*(*x*, *t*) which denote the population of the prey and predator, respectively, in a single patch. The solutions predict the two following behaviors

### 4.1. The (*G*′/*G*)-Expansion Method (Solution (1))

As a result of two predators' sexual interaction and the high prey consumption during the predator's mating period, *V* increases and *U* decreases. Ultimately, *V* will become dominant in the patch.

### 4.2. Generalized Auxiliary Equation Method (Solution (2))

The predators graze in the mating period where the prey density (*U*) is large. Then, *U* decrease and *V* increase. At a certain time, *U* will be very low, and the predators will either die or move to different patches. Then, the prey population will recover and grow again in the same location.

### 4.3. Exponential Time Differencing Method

For a large value of *k*_2_, we obtain the numerical solution that converges to solution (1), while for small *k*_2_, the numerical solution approximates solution (2).

The numerical solution gives the important reasons behind the two different solutions by the analytical methods.

## 5. Conclusion

The prey-predator system with the extra term *a*_4_*v*^2^*u* (1) is a new nonlinear dynamic system of equations in the literature. It has been solved analytically with two different methods which give two different solutions. The importance of this paper is that the numerical solution gives connection between the obtained analytical solutions from the biological perspective. The numerical solution predicts the dynamic of the studied model as well as proves the effect of the new extra term on the model.

## Figures and Tables

**Figure 1:** Plot of *U*, *V* for *k*_1_ = 1 and $0<k_{2}<\left(1+\sqrt{5}\right)/2.$

**Figure 2:** Plot of *u*, *v* for *a*_1_ = *a*_2_ = 1, *a*_5_ = 0.5 to capture the effect of the term *a*_4_*uv*^2^ on the model.

**Figure 3:** Plot of *u*, *v* for *a*_1_ = *a*_2_ = 1, *a*_5_ = 0.5 to capture the effect of the term *a*_3_*uv* on the model.

## Data Availability

The data supporting this research are from previously reported studies, which have been cited.
